# Ticks and associated pathogens in dogs from Greece

**DOI:** 10.1186/s13071-017-2225-2

**Published:** 2017-06-23

**Authors:** Maria Stefania Latrofa, Athanasios Angelou, Alessio Giannelli, Giada Annoscia, Silvia Ravagnan, Filipe Dantas-Torres, Gioia Capelli, Lenaig Halos, Frederic Beugnet, Elias Papadopoulos, Domenico Otranto

**Affiliations:** 1 Dipartimento di Medicina Veterinaria, Università degli Studi di Bari, Valenzano, Bari, Italy; 2 School of Veterinary Medicine, Faculty of Health Sciences, Aristotle University of Thessaloniki, Thessaloniki, Greece; 3 Istituto Zooprofilattico Sperimentale delle Venezie, Legnaro, Padua, Italy; 4 Departamento de Imunologia, Instituto de Pesquisas Aggeu Magalhães (Fiocruz-PE), Recife, Pernambuco Brazil; 5 Merial SAS (Boehringer Ingelheim), 29 avenue Tony Garnier, Lyon, France

**Keywords:** Ticks, Tick-borne pathogens, Dogs, Greece, PCR, qPCR, TBDs

## Abstract

**Background:**

With the aim to assess the occurrence of hard ticks and the pathogens they may carry in dogs from Greece, ixodid specimens (*n* = 757) were collected from 310 animals living in six provinces across the Greek peninsula. All ticks were morphologically identified, and genomic DNA was extracted from 344 (45.5%) representative specimens, according to their species, engorgement status and sampling area. The occurrence of *Anaplasma* spp., *Ehrlichia* spp., *Hepatozoon* spp., *Rickettsia* spp., *Babesia* spp., *Theileria* spp. and *Cercopithifilaria* spp. was assessed by conventional and quantitative real-time PCR.

**Results:**

Overall, 150 dogs (48.4%) were infested by ticks, with *Rhipicephalus sanguineus* (*sensu lato*) being the most prevalent (70.1%), followed by *Haemaphysalis parva* (14.7%), *Rhipicephalus turanicus* (11.4%), and *Haemaphysalis concinna* (2.4%). Out of 344 specimens molecularly examined, 41 (11.1%) were positive for at least one microorganism (i.e. 5.5% for *Cercopithifilaria bainae*, 2.9% for *Hepatozoon canis*, 1.7% for *Rickettsia hoogstraalii*, 1.2% for *Hepatozoon felis*, 0.6% for *Rickettsia massiliae*, 0.6% for *Theileria ovis*, 0.3% for *Anaplasma platy*s and 0.3% for *Coxiella* like-endosymbiont).

**Conclusions:**

The results of this study show that different tick species parasitize dogs in Greece, carrying a range of microorganisms potentially pathogenic for dogs and humans. Consequently, control strategies against ticks are of great importance to prevent the risk of tick-borne diseases. The relationship between ticks infesting dogs and associated microorganisms is described according to collection site and dog lifestyle.

## Background

Ticks represent a major threat to domestic and wild animals worldwide due to blood depletion, inoculation of toxins and allergens and, importantly, pathogen transmission [1]. A range of viruses, bacteria and protozoa causing tick-borne diseases (TBDs) induces economic losses in livestock production [2] and puts at risk the health of companion animals [3, 4]. In addition, several tick-borne pathogens are of zoonotic concern and their transmission to humans is related to a number of driving factors, including the presence of proper vectors and hosts [5–8]. The distribution of ticks and their vectored pathogens is affected by a plethora of biological and environmental determinants, including climate changes, deforestation, and urbanisation, which may together favour the spreading and establishment of selected vectors into previously free areas [9–11]. The scientific knowledge on the ecology of different tick species becomes, therefore, pivotal to assess the risk factors for pathogen transmission.

The Mediterranean basin provides an optimal environment for the development of a number of tick species [12–14]. In Greece, for instance, a range of ixodid species has been reported in domestic animals and humans, including *Rhipicephalus sanguineus* (*sensu lato*), *Rhipicephalus turanicus*, *Rhipicephalus bursa*, *Hyalomma marginatum*, *Hyalomma rufipes*, *Hyalomma turanicum*, *Hyalomma excavatum*, *Hyalomma scupense*, *Ixodes ricinus*, *Ixodes gibbosus*, *Ixodes hexagonus*, *Haemaphysalis inermis*, *Haemaphysalis punctata*, *Haemaphysalis sulcata*, *Haemaphysalis parva*, *Dermacentor marginatus* and *Amblyomma variegatum* [15–20].

While most of the studies carried out have focused their attention on the ixodid fauna of livestock, only a few have been performed on dogs, mainly in the northern part of the Greek peninsula [16, 17]. Accordingly, selected canine tick-borne pathogens (e.g. *Hepatozoon canis*, *Anaplasma* spp., *Rickettsia* spp. and *Cercopithifilaria* spp.) have also been detected [21–23], although there is no clear association between tick species and their pathogens.

In order to fill this gap in knowledge, this study aimed to investigate the distribution of hard ticks and carried pathogens in dogs living under different conditions across Greece.

## Methods

### Tick collection and identification

From May to August 2015, tick specimens were collected on domestic dogs living in six provinces across Greece (Fig. 1, Table 1), specifically from southern (Corinth, site A; Athens, site B), central (Larisa, site C) and northern regions (i.e. Xanthi, site D; Thessaloniki, site E; Alexandroupoli, site F). Ticks were sampled on animals from rural areas, municipal shelters, temporary kennels, indoor environments, or in hospitalised animals (Table 1).

**Fig. 1:** Distribution of tick species and their positivity for microorganisms according to the sampling site

**Table 1:** Area and provinces of Greece surveyed, along with information of infested dogs according to sampling site (A-F) and tick developmental stages

Area	Province	Dogs						Ticks					
		Rural areas	Indoors	Temporary kennel	Municipal shelter	Private clinics	Infested dogs (%)	Larvae	Nymphs	Adults		Total specimens collected	Intensity
										Male	Female		
Southern	Corinth (A)	8/12	10/18	12/12	0/4	0/4	30/50 (60)	–	33	50	60	143	4.77
	Athens (B)	0/2	10/30	–	10/25	0/23	20/80 (25)	–	16	26	30	72	3.5
Central	Larisa (C)	5/10	5/12	10/10	0/2	0/6	20/40 (50)	–	19	13	19	48	2.6
Northern	Xanthi (D)	24/28	–	–	0/2	6/10	30/40 (75)	3	224	11	23	261	8.8
	Thessaloniki (E)	4/6	5/21	17/17	14/22	0/14	40/80 (50)	23	57	28	93	201	5.0
	Alexandroùpolis (F)	0/1	2/3	–	8/14	0/2	10/20 (50)	2	6	16	5	29	2.8
Total (%)		41/59 (69.5%)	32/84 (38.1%)	39/39 (100%)	32/69 (46.4%)	6/59 (10.2%)	150/310 (48.4%)	28 (3.7%)	355 (46.9%)	144 (19%)	230 (30.4%)	757	

All ticks were preserved in 70% ethanol and categorised according to their gender and developing stages. Specimens were morphologically identified at species level using morphological keys [12, 24, 25].

### Pathogen molecular diagnosis

Genomic DNA was extracted from a representative number of tick specimens, according to their species, engorgement status and sampling area. Ticks were cut into small pieces using sterile scalpels, homogenized in 300 μl of DNA extraction buffer (20 mM Tris-HCl pH 8; 100 mM EDTA and 1% SDS, 400 μg proteinase K), and incubated overnight at 37 °C. Protein was precipitated using 50 μl of 5 M potassium acetate, before samples were stored on ice for 10 min and centrifuged at 13,000× *g* for 5 min. The DNA pellet was precipitated using 300 μl of 100% isopropanol followed by centrifugation at 13,000× *g* for 5 min and a final wash with 300 μl of 70% ethanol and centrifugation at 13,000×*g* for 5 min. Pellets were air dried and resuspended in 50 μl TE (10 mM Tris-HCl, 1 mM EDTA pH 8).

Target sequences of *Anaplasma*/*Ehrlichia* spp., *Babesia*/*Theileria* spp. and *Rickettsia* spp. were detected by quantitative real-time PCR assays (qPCR), as described previously [26–28]. In addition, DNA of canine filarioids and *Hepatozoon* spp. was detected by conventional PCR amplification of partial cytochrome *c* oxidase subunit 1 (*cox*1, 690 bp) and 18S rRNA (~670 bp) genes, respectively, using primers and cycling protocols described previously [29, 30].

PCR products were examined on 2% agarose gels stained with GelRed (VWR International PBI, Milano, Italy) and visualised on a GelLogic 100 gel documentation system (Kodak, New York, USA). The amplicons were purified and sequenced in both directions using the same primers used for PCR and qPCR, employing the Big Dye Terminator v.3.1 chemistry in a 3130 genetic analyser (Applied Biosystems, California, USA). Sequences were aligned using the ClustalW program [31] and compared with those available in GenBank by Basic Local Alignment Search Tool (BLAST - http://blast.ncbi.nlm.nih.gov/Blast.cgi).

### Statistical analysis

Prevalence (proportion of hosts infested by ticks and of tick species positive for a given pathogen) and tick infestation burden (arithmetic mean count of ticks on each infested hosts) were assessed. For prevalence rates > 5%, Fisher’s exact test was used to compare the prevalence of infection among sampling areas, and among dog keeping conditions. Differences were considered significant when *P* <0.05. Statistical analyses were performed using BioEstat 5.0.

## Results

Of the 310 dogs examined, 150 (48.4%) harboured ticks, with the infestation prevalence varying according to sampling sites and dog keeping conditions (Table 1). Out of 757 ticks collected, 374 (49.4%) were adults (i.e. 230 females and 144 males), 355 (46.9%) nymphs and 28 (3.7%) larvae.

Overall, four tick genera and seven species were identified (Table 2), with the most representative tick species being *R. sanguineus* (*s*.*l*.) (70.1%), followed by *H. parva* (14.7%), *R. turanicus* (11.4%) and *H. concinna* (2.4%) (Fig. 1, Table 2). Mixed infestations were recorded in 10 dogs (6.7%), three of which harboured *H. parva* and *H. concinna*, two *H. parva* and *R. sanguineus* (*s*.*l*.) or *H. parva* and *I. ricinus*, and one each *Hyalomma scupense* and *R. bursa*, *R. sanguineus* (*s*.*l*.) and *R. turanicus*. One dog was simultaneously infested by *H. parva, R. sanguineus* (*s*.*l*.) and *I. ricinus.*

**Table 2:** Tick species, with their intensity (ticks on infested animals) and microorganisms detected according to collection sites and developmental stage. Ticks positive for pathogens are reported in bold

Tick species	Number of ticks	Intensity	Collection site/number of ticks	Microorganism (positive/ticks tested) and tick developmental stage							
				*Cercopithifilaria bainae*	*Hepatozoon canis*	*Hepatozoon felis*	*Anaplasma platys*	*Rickettsia hoogstraalii*	*Rickettsia massiliae*	*Theileria ovis*	*Coxiella*-like endosimbiont
*Haemaphysalis concinna*	18	2.6	C/6	0/3	**1/3 M** ^**c**^	0/3	0/3	0/3	0/3	0/3	0/3
			E/6	0/3	**1/3 M** ^**c**^	0/3	0/3	0/3	0/3	0/3	0/3
			F/6	0/2	0/2	0/2	0/2	0/2	0/2	0/2	0/2
			C/6	0/3	**1/3 M** ^**c**^	0/3	0/3	0/3	0/3	0/3	0/3
			E/6	0/3	**1/3 M** ^**c**^	0/3	0/3	0/3	0/3	0/3	0/3
			F/6	0/2	0/2	0/2	0/2	0/2	0/2	0/2	0/2
*Haemaphysalis parva*	111	3.8	C/20	0/17	0/17	**1/17 M** ^**c**^	0/17	**1/17 M** ^**c**^	0/17	0/17	0/17
			E/84	**2/39 F** ^**c**^	**2/39 F** ^**c**^	0/39	0/39	**5/39 F** ^**c**^	0/39	0/39	0/39
			F/7	0/5	0/5	0/5	0/5	0/5	0/5	0/5	0/5
*Haemaphysalis* spp.	2	–	F/2	0/1	0/1	0/1	0/1	0/1	0/1	0/1	0/1
*Hyalomma scupense*	1	–	D/1	0/1	0/1	0/1	0/1	0/1	0/1	0/1	0/1
*Ixodes ricinus*	2	–	E/2	0/1	0/1	0/1	0/1	0/1	0/1	0/1	0/1
*Rhipicephalus bursa*	1	–	D/1	0/1	0/1	0/1	0/1	0/1	0/1	**1/1 M** ^**a**^	0/1
*Rhipicephalus sanguineus* (*s.l*.)	531	5.2	A/127	**3/51 N** ^**a**^	0/51	**1/51 N** ^**a**^	0/51	0/51	0/51	0/51	0/51
			B/69	**3/37 F** ^**b**^	**2/37 N** ^**d**^	**1/37 N** ^**b**^	0/37	0/37	0/37	0/37	**1/37 F** ^**b**^
			C/25	0/15	0/15	**1/15 F** ^**b**^	0/15	0/15	0/15	0/15	0/15
			D/221	**4/79 F** ^**a**^	0/79	0/79	0/79	0/79	0/79	**1/79 M** ^**d**^	0/79
			E/75	**2/39 N** ^**c**^	**2/39 F** ^**d**^	0/39	**1/39 N** ^**b**^	0/39	**1/39 L** ^**d**^	0/39	0/39
			F/15	**2/13 L** ^**a**^	**1/13 L** ^**a**^	0/13	0/13	0/13	0/13	0/13	0/13
*Rhipicephalus turanicus*	86	4.5	A/16	**1/5 N** ^**a**^	**1/5 N** ^**a**^	0/5	0/5	0/5	0/5	0/5	0/5
			B/3	0/2	0/2	0/2	0/2	0/2	0/2	0/2	0/2
			D/38	0/10	0/10	0/10	0/10	0/10	0/10	0/10	0/10
			E/29	**2/18 N** ^**d**^	0/18	0/18	0/18	0/18	**1/18 N** ^**d**^	0/18	0/18
*Rhipicephalus* spp.	5	2.5	E/5	0/2	0/2	0/2	0/2	0/2	0/2	0/2	0/2
Total (%)	757	3.7		19/344 (5.5)	10/344 (2.9)	4/344 (1.2)	1/344 (0.3)	6/344 (1.7)	2/344 (0.6)	2/344 (0.6)	1/344 (0.3)

^a^ Rural area

^b^ Indoor

^c^ Temporary kennel

^d^ Municipal shelter

*Abbreviations*: L, larva; N, nymph; M, male; F, female

*Legend*: A, Corinth; B, Athens; C, Larisa; D, Xanthi; E, Thessaloniki; F, Alexandroùpolis

Ticks positive for pathogens are reported in bold

Though not statistically significant (*P* > 0.05), the tick burden varied according to dog type (i.e. dogs sheltered in temporary kennels or living in rural areas were more often infested than those referred to private veterinary clinics or housed indoor) and the sampling sites. Dogs from site D (northern Greece) harboured more ticks than those from sites B and C (southern and central Greece) (Table 1). While *R. sanguineus* (*s*.*l*.) was found in all the sampling areas, *R. turanicus* and *H. parva* were not detected in site C and sites A, B or D, respectively (Table 2). Specimens of *I. ricinus*, *H. scupense* and *R. bursa* were found only in northern regions (Fig. 1, Table 2). *Rhipicephalus sanguineus* (*s*.*l*.), *R. turanicus*, *R. bursa* and *H. scupense* were thoroughly collected from dogs living in rural areas, municipal shelter, and referred to private clinics, whereas *Haemaphysalis* spp. were mainly found on animals from temporary kennels (Table 2).

Out of 344 specimens analysed, 41 (11.1%) were positive for at least one microorganism based on PCR (Table 2), with the largest number of positives being detected in the northern regions (Fig. 1). Nineteen ticks (5.5%; nine females, two larvae, and eight nymphs) were positive for *Cercopithifilaria bainae*, 10 (2.9%; two males, four females, one larva, and three nymphs) for *H. canis* and six (1.7%; one male and five females) for *Rickettsia hoogstraalii*. Other microorganisms were detected less frequently, such as *Hepatozoon felis* (1.2%; one male, one female, and two nymphs), *Rickettsia massiliae* (0.6%; one larva and one nymph), *Theileria ovis* (0.6%; two males), *A. platy*s (0.3%; one nymph) and for a *Coxiella*-like-endosymbiont (0.3%; one female) (Table 2, Fig. 1). Co-infections with multiple microorganisms were detected in six specimens. In particular, *C. bainae* was detected in combination with *H. felis* or *H. canis* or *R. massiliae* in *R. sanguineus* (*s*.*l*.), and with *H. canis* in *R. turanicus*. *Rickettsia hoogstraalii* was simultaneously diagnosed with *H. felis* or *H. canis* and *C. bainae* in *H. parva*. Associations between tick developmental stages, dog lifestyles, collection site and microorganisms are reported in Table 2, and none of the parameters evaluated was statistically significant (*P* > 0.05).

BLAST analysis confirmed the identification of the detected microorganisms with the highest nucleotide identity of 98–100% with the sequences available in the GenBank database (Accession numbers: KF270686, AJ537512, KC138534, KJ605146, KJ605147, EF201806, KX273858, KJ663754, EF629536).

## Discussion

Data from this study indicate that dogs from Greece are exposed to different tick species and, potentially, to several tick-borne pathogens, whose occurrence is not strictly influenced by the conditions in which dogs live. Nonetheless, the finding of a higher tick burden in animals from kennels, rural areas or municipal shelters compared to those kept indoor is presumably related to the frequency of treatment against ectoparasites, which is performed more frequently in pet than in shepherd or kennelled dogs [32].

Overall, the collection of different tick species in each of the geographical areas confirms the existence of a marked ixodid diversity in the Greek peninsula [16, 20, 22] with a higher number of ticks sampled in northern areas bordering continental Europe (i.e. Macedonia, Turkey and Albania) [16, 32, 33] than southern regions [16, 20].

*Rhipicephalus sanguineus* (*s*.*l*.) was the most prevalent species throughout Greece, most likely due to its strict affiliation to canids [25], and/or its ability to survive in a large array of environmental conditions [13, 16, 34–36]. Conversely, the finding of *R. turanicus* on dogs is probably related to its adaptability to several vertebrate animals, including goats and sheep [25], which have a major role in the economy of this country. Along with *R. bursa* and *H. scupense*, *R. turanicus* can often be detected on livestock in the northern regions of Greece [20], where they often parasitize dogs [16]. *Haemaphysalis parva* and *H. concinna* usually parasitize birds as larvae and nymphs, and herbivores as adults [24]. Finding these species on dogs was likely due to the location of animal shelters, close to forested, meadow and rural habitats [37].

Amongst the microorganisms detected, the filarioid *C. bainae* was the most common, being found in *R. sanguineus* (*s*.*l*.), as previously reported [22]. The detection of *C. bainae* in *H. parva* probably occurred during the ingestion of skin-dwelling microfilariae during the tick blood meal. Nonetheless, considering that the same tick species was found positive for *H. canis* and *H. felis*, its implication as a vector for these pathogens cannot be ruled out. Though *H. felis* has been detected in *R. sanguineus* (*s*.*l*.) [38, 39], the vector of this protozoon remains unknown, whereas *H. canis* has been so far been detected in a number of other tick species, including *Haemphysalis* spp. and *R. turanicus* [40, 41]. In the current study, *H. parva* specimens were positive for *R. hoogstraalii*, adding new scientific information to knowledge on this *Rickettsia* species. *Rickettsia hoogstraalii* was originally isolated from *H. sulcata* from sheep and goats in Croatia [42], *H. punctata* and *H. sulcata* from Spain [43] and, in the same tick species from foxes in Cyprus [44]. *Rickettsia massiliae* was here found in *R. sanguineus* (*s*.*l*.) and *R. turanicus* collected from dogs living in municipal shelters in northern Greece, close to the Turkish boundaries. This finding is not surprising when considering that the transstadial and transovarial transmission of *R. massiliae* has been described in both *Rhipicephalus* species [45]. Besides the current report, *R. massiliae* has been detected in *R. sanguineus* (*s*.*l*.) and *R. turanicus* from Greece and other countries (e.g. Spain, Portugal, Switzerland, France, Algeria, Morocco, Israel and Italy) [6, 46], as well as in *Rhipicephalus mushamae*, *Rhipicephalus lunulatus*, *Rhipicephalus sulcatus* and *Rhipicephalus guilhoni* [6, 25].

Remarkably, *R. massiliae* has not yet been isolated from humans in Greece, but its detection in *Rhipicephalus* spp. ticks suggest that the risk for human infections is probably underestimated [46, 47]. The absence of *E. canis* and *Babesia vogeli* positive ticks in this study was surprising as both pathogens are transmitted by *R. sanguineus* (*s*.*l*.) ticks [48, 49], and could be explained by their transitory parasitaemia and by the number of ticks examined.

## Conclusions

The results of this study show that different tick species parasitize dogs in Greece, carrying a range of microorganisms potentially pathogenic for dogs and humans. As such, control strategies against ticks are of great importance to prevent the risk of TBDs.

## Abbreviations

*cox*1: Cytochrome *c* oxidase subunit 1
qPCR: quantitative real-time PCR assays
TBDs: Tick-borne diseases
